# Study on the Relationship between lncRNA Gene Polymorphism and Systemic Lupus Erythematosus

This article has been retracted.

**DOI:** 10.1155/2022/4446016

**Published:** 2022-02-27

**Authors:** Xue Guan, Dan Liu, Yuling Xing, Xiuru Guan

**Affiliations:** ^1^Clinical Laboratory, First Affiliated Hospital of Harbin Medical University, 150001, China; ^2^Clinical Laboratory, Qingdao Hospital of Traditional Chinese Medicine (Qingdao Hiser Hospital), 266033, China

## Abstract

**Background:**

Systemic lupus erythematosus (SLE) is an autoimmune disease that can cause damage to multiple systems of the body. A number of studies have shown that long-chain noncoding RNA (lncRNA) can participate in the occurrence and development of a variety of autoimmune diseases. This study is aimed at detecting the expression levels of 5 lncRNAs in SLE patients and healthy controls and at exploring the relationship between expression levels and clinical symptoms and laboratory indicators.

**Methods:**

The design type of this study is a case-control study. A total of 76 SLE patients and 71 healthy controls were included in the first phase of the study. Real-time fluorescence quantitative polymerase chain reaction was used to detect the expression level of 5 kinds of lncRNAs including lnc7514, lnc0640, lncagf, nc3643, and lnc5150 in PBMCs of two groups of patients; the expression of lncRNAs in the case group and the control group was analyzed. We analyzed the differences in the expression levels of lncRNAs between case and control groups, and explored the association of expression levels with clinical manifestations and laboratory characteristics. SPSS23.0 was used to analyze the expression level and gene polymorphism results; the statistical analysis test level *α* = 0.05.

**Results:**

The expression level of lnc0640 in PBMCs of SLE patient group was higher than that of healthy control group (*Z* = −3.56, *P* = 0.03). However, lnc5150 was lower than in healthy controls (*Z* = −7.16, *P* < 0.001). lnc3643 expression levels were lower in SLE patients of SLE patients with pleurisy was lower than that of patients without pleurisy (*Z* = −2.44, *P* = 0.02). Low lnc3643 expression levels were observed in PBMCs with SLE patients with rash symptoms (*Z* = −2.75, *P* = 0.013). SLE expressed lower lnc3643 levels in PBMCs with SLE compared with those without pleurisy (*Z* = −2.42, *P* = 0.02). The above differences were statistically significant. Association analysis of lncRNA expression levels and clinical manifestations in SLE patients found that SLE was lower than those without rash or pleurisy (both *P* < 0.05); association analysis of lncRNA expression level and laboratory results found a negative correlation between lnc3643, lnc7514, and SLE disease activity score (SLEDAI-2K), blood sink (ESR), and C-reactive protein (CRP) (all *P* < 0.05).

**Conclusions:**

lnc0640 was overexpressed in PBMCs in SLE patients compared with healthy controls. lnc3643 was negatively correlated with SLEDAI, and expression levels were associated with SLE patients with arthritis, rash, and pleuritis.

## 1. Introduction

Systemic lupus erythematosus (SLE) is a common autoimmune disease that can lead to irreversible damage to the body's immune tolerance [1, 2]. Because clinical heterogeneity leads to different clinical manifestations and outcomes in SLE patients, clinical heterogeneity makes no certain single detection method available to confirm SLE [3]. Studies have shown that the etiology of SLE may be environmental factors, genetic factors, and hormones and interactions and that genetic factors may play a key role in the pathogenesis of SLE [4, 5].

The genetic background of SLE mainly includes encoding genes and noncoding genes (nRNA), while nRNA can be divided into short-chain nRNA and long-chain nRNA (lncRNA) based on the length size [6]. lncRNA is a class of endogenous RNA molecules with >200 bp in length and has no protein-coding function [7]. It has been found that lncRNA can bind to DNA, RNA, or proteins to form complexes to regulate gene activation and transcriptional processes, and some lncRNAs can even encode small functional polypeptide chains [8].

Previous studies found that lnc0597 and lnc0949 expression was lower in peripheral blood mononuclear cells (PBMCs) in SLE patients than in healthy populations, lower lncRNA GAS5 and lnc-DC in SLE plasma than in healthy controls, and higher lnc0597 levels than in healthy populations [9, 10]. In addition, more studies have also shown lncRNA involvement in the occurrence and development of autoimmune diseases [11, 12]. This study is aimed at exploring the role of lncRNAs in the occurrence and development of SLE and at providing evidence for further exploration of SLE markers and therapeutic targets.

## 2. Data and Methods

This experiment was designed as a case-control study, using quantitative reverse transcriptase chain reaction (qRT-PCR) technology was used to detect the expression levels of lncRNA in PBMCs in SLE patients and healthy controls and explore the correlation of lncRNA expression with the main clinical symptoms of SLE and laboratory testing indicators. See Figure 1 for the experimental flow chart.

### 2.1. Subject Investigated

#### 2.1.1. Selection of Patients with SLE

*Patient inclusion criteria for this study*: According to the SLE classification criteria revised by the American College of Rheumatology (ACR) as the basis for the diagnosis of SLE cases, those who meet the diagnosis can be included. Diagnostic criteria are shown in Table 1. *Exclusion criteria*: (1) patients with other autoimmune diseases; (2) combined systemic infected persons; (3) patients with severe heart, liver, and renal failure; (4) patients with other malignant tumors, neurodegenerative diseases, and mental diseases; and (5) unwilling to participate in the investigation. Patients diagnosed with SLE and not having any feature of the exclusion criteria could be included in this study.

#### 2.1.2. Selection of Healthy Controls

Healthy controls were obtained from 71 healthy patients in the physical examination center of the hospital. The selected pairs should meet the following criteria: no history of autoimmune disease, any of the annual SLE classification criteria, immediate relatives with no history of autoimmune disease, and no hormones and immunosuppressants for the last month.

During the clinical classification and diagnosis process, patients meet the above four criteria before or after the onset and can be diagnosed as SLE after excluding tumor, infection, and other connective tissue disease.

### 2.2. Collection of Data and Samples

#### 2.2.1. Questionnaire

Trained investigators communicate with patients meeting SLE screening criteria and with informed consent, and a unified data collection was used to design the questionnaire. The SLE questionnaire mainly includes general information (name, gender, education, contact information, etc.), clinical data (major clinical symptoms, disease course, clinical medication, etc.), and laboratory indicators (anti-ds-DNA, anti-Sm, anti-SSA/Ro, anti-SSB/La, anti-RNP, anti-Ribosomal P, C3, C4, ESR, CRP, etc.), and patient disease activity was evaluated according to the SLE disease activity score scale. General demographic data (name, gender, age) were collected from healthy controls.

#### 2.2.2. The Quality Control of Questionnaire

(1) The quality of the questionnaire determines the quality of the survey results; preinvestigation is required to evaluate the feasibility, authenticity, and validity of the questionnaire after review by experts and reference to literature and for timely revision; (2) for the graduate students who participated in the questionnaire, carry out prejob training, unify the investigators' understanding of the meaning of the survey indicators, clarify the purpose of the survey, and master the survey skills; (3) register and verify the collected questionnaire data, correspond the blood samples, and supplement the missing information in a timely manner. Ensure the integrity of the questionnaire.

#### 2.2.3. Specimen Collection

5 ml of peripheral venous blood was selected in anticoagulant vessels containing ethylenediaminetetraacetic acid (EDTA). The extracted blood samples were added to the lymphocyte isolate for 4 h to separate the lymphocytes, and the total RNA was extracted and stored in the -80 C refrigerator.

#### 2.2.4. Detection of Samples

The expression levels of lnc0640, lnc3643, lnc5150, lnc7514, and lncagf were subjected to the lnc0640, lnc3643, lnc5150, and lncagf by real-time polymerase chain reaction (qRT-PCR). The detection procedure is shown in Figure 2.

#### 2.2.5. Arrangement and Entry of Data

(1) Make a one-to-one number of the questionnaire and blood samples, (2) check and logically check the questionnaire and experimental data results to ensure the authenticity and accuracy of the original data, and (3) use EpiData 3.1 double input and error detection mode into the questionnaire.

### 2.3. Statistical Analysis

(1) In the detection of lncRNAs content, 2−△△Ct is used to represent the relative expression level of the target gene (Ct: the number of cycles experienced when the amplification product of the target gene or parameter reaches the set threshold; △Ct: mean Ct value of target gene-mean Ct value of the reference gene). (2) EpiData 3.1 was used for double entry of experimental data, and SPSS 23.0 software was used for data analysis. (3) Quantitative data meeting the normal distribution are described using (*x* ± *s*); quantitative interdata comparisons were performed using *t*-test/ANOVA statistics; M(P25, P75) was used to describe the quantitative data that did not conform to the normal distribution, and the Mann–Whitney rank-sum test was used for the comparison between the data; the 2 tests were used for the qualitative data comparison. In the correlation analysis between the two groups, the two groups' samples were normal. Pearson's correlation was used for distribution, and Spearman's rank correlation was used when a group of samples did not conform to normal distribution. Statistical analysis of sex and age and gene sites before and after correction was analyzed by logistic regression; gene polymorphism results were analyzed using *Z* test, with test level =0.05.

## 3. Results

### 3.1. General Data of Both Patient Groups

We collected 76 SLE patients and 71 in the healthy control group; 69 (90.8%) women in the case group and 7 (9.2%) men; and 62 (87.3%) women in the control group and 9 (12.7%) men. The mean age in the case group was 37.54 ± 9.68 years, and the median age in the control group was 39.32 ± 5.32 years. The average disease course of SLE patients was 2.21 ± 4.26 years, and the average SLEDAI score was 12.60 ± 3.07. Basic data were not statistically significant in both groups (*P* > 0.05) (see Table 2).

### 3.2. lncRNA Expression Level

lnc0640 expression levels were higher in SLE than in healthy controls (HC) (*Z* = −2.23, *P* = 0.03), while lnc5150 was lower in SLE than in HC (*Z* = −6.02, *P* = 0 < 0.001), and the remaining genes between SLE and healthy controls (see Figure 3).

### 3.3. Analysis of the Association between lncRNA Expression Level and Clinical Manifestations in SLE Patients

SLE patients were divided into groups according to whether they had arthritis, rash, myositis, pleurisy, fever, and other clinical manifestations. Mann–Whitney rank-sum test was used to compare the differences in the expression levels of five lncRNAs among subgroups. The difference was statistically significant (*Z* = −2.44, *P* = 0.02). The lnc3643 expression levels were low in PBMCs of patients with SLE with rash symptoms compared with patients with no rash symptoms. The level difference between the two groups was statistically significant (*Z* = −2.75, *P* = 0.01); SLE with SLE expressed lower PBMCs in SLE compared with those without pleurisy, and the difference was statistically significant (*Z* = −2.42, *P* = 0.02). The expression levels of lncRNAs were different between myositis and febrile subgroups. However, the difference was not significantly significant (all with *P* > 0.05) (see Table 3).

### 3.4. Analysis of the Correlation between the Expression Level of lncRNAs and Laboratory Indicators in SLE Patients

Mann–Whitney rank-sum test is shown in Table 4. The results showed that lnc7514 expression levels were lower in dsDNA (+) than in dsDNA (-), significant (*Z* = −2.70, *P* = 0.01), SSA (+), negative (*Z* = −2.381, *P* = 0.017). lncagf expression levels are between different groups of RNP (*Z* = −2.01, *P* = 0.05); there is no association of the expression levels of laboratory indicators Sm and SSB (all *P* > 0.05).

### 3.5. Analysis of the Correlation between lncRNA Expression Level and SLE Disease Activity

Spearman rank correlation was used to analyze the correlation between lncRNA expression levels and complement C4 levels, blood sink (ESR) levels, SLEDAI score, C-reactive protein (CRP) levels, and course of disease, as shown in Table 5. The lnc3643 expression levels were negatively correlated with the levels of ESR, CRP, and SLEDAI (rs = −0.46, *P* < 0.001; rs = −0.42, *P* < 0.001; rs = −0.25, *P* = 0.03). lnc5150 expression levels were negatively correlated with ESR levels (rs = −0.39, *P* = 0.01). The expression levels of lnc7514 were negatively correlated with the levels of ESR, CRP, and SLEDAI (rs = −0.38, *P* < 0.001; rs = −0.25, *P* = 0.03; rs = −0.31, *P* = 0.01). The level of lncagf expression was also negatively correlated with ESR levels (rs = −0.27, *P* = 0.02). No association was found between lnc0640 expression levels and each disease activity index (all with *P* > 0.05).

## 4. Discussion

SLE is an autoimmune disease with a complex etiology and with a genetic tendency and familial aggregation [13]. Recent studies have found that lncRNA can be involved in many cellular functional processes, such as gene imprinting, functional protection, lineage submission, and apoptosis [14]. It has also been shown that lncRNAs can be involved in the development of autoimmune diseases such as SLE, rheumatoid arthritis, and scleroderma [15, 16]. Identifying the role of lncRNAs in SLE disease contributes to the better diagnosis and treatment of SLE disease.

In this study, the relationship between five lncRNAs and SLE, including lnc0640, lnc3643, lnc5150, lnc7514, and lncagf, were explored. It mainly investigated the differences in lncRNA expression levels between SLE and healthy controls and explored the relationship between lncRNA expression levels and clinical symptoms, laboratory examination, etc. Previous studies found higher plasma levels of lnc0640 in SLE patients than in healthy controls and that lnc5150 was upregulated in PBMCs compared with healthy controls [17, 18].This study found higher lnc0640 expression levels in PBMCs in the SLE patient group compared with healthy controls, which is consistent with the above study. However, the results of this study found that lnc5150 has lower expression in SLE patients, probably due to intracellular to extracellular release through efflux, leading to higher extracellular lnc5150 levels than in the normal state. In addition, this study found a negative correlation of lnc5150 expression levels with ESR levels. The above results suggest that lnc5150 may be associated with the occurrence and development of SLE.

In this study, a study in SLE with symptoms found that lnc3643 expression levels were lower in PBMCs of patients with rash or pleurisy than in those without this clinical symptom, and association analysis studies found inverse expression levels of ESR, CRP, SLEDAI, and lnc3643. The above results suggest that lnc3643 may be related to the occurrence of SLE inflammation and that lnc3643 may be used as an indicator to monitor SLE condition and guide treatment, which needs further investigation.

lnc7514 and lncagf expression levels did not differ in SLE patients and healthy controls, further research on the relationship between clinical symptoms and laboratory test results in SLE patients found that the expression level of lnc7514 decreased in patients with anti-dsDNA and lnc7514 was inversely associated with ESR, CRP, and SLEDAI, suggesting that lnc7514 may be related to the occurrence of SLE inflammation and disease activity. The expression levels of lncagf were downregulated in patients with anti-SSB and anti-RNP compared with those without two laboratory examinations and were negatively correlated with ESR.

The feature and innovation of this study is that it is the first time to investigate the expression of lnc0640, lnc3643, lnc5150, lnc7514, and lncagf genes and their association with clinical characteristics in Chinese Han population. However, this study also has some limitations. First, this study was a hospital-based case-control study with selection bias and confounding bias. Second, fewer subjects in this experiment failed to analyze the association between expression level and gene polymorphism. Moreover, due to the related problems of department management, no patients were included in this study. It is hoped that the subsequent experimental research can make up for the above shortcomings, further explore the association of genetic loci and genetic susceptibility to SLE more deeply, and provide strong evidence for the study of this gene in other diseases or populations.

## 5. Conclusion

1. Compared to normal controls, the expression levels of lnc3643, lnc7514, and lncagf in PBMCs in SLE patients may not be associated with SLE occurrence, while lnc0640 and lnc5150 expression levels may be associated with SLE occurrence
2. lnc0640 and lnc5150 had no association with genetic susceptibility to SLE; lnc3643 expression levels were associated with arthritis, rash, and SLE pleuritis

## Figures and Tables

**Figure 1:** Experimental flow.

**Figure 2:** The main process of lncRNA expression level detection.

**Figure 3:** Comparison of the expression levels of lncRNAs between cases and controls.

**Table 1:** Diagnostic criteria for SLE.

Group standard	Definition of relevant indicators
Face butterfly red spot	Flat or higher throughout the neck than the skin fixed erythema, often does not involve the nasal and labial groove site
Discal red spots	The bulge erythema is covered with keratin scales and hair follicle damage, and there can be atrophic scar on the old lesions
Daylight allergy	Sunlight exposure causes an abnormal skin reaction and produces a rash
Dental ulcer	Painless ulcer in the mouth or nasopharyngeal
Arthritis	Nonerosive arthritis, involving 2 or more peripheral joints, must have inflammatory manifestations (e.g., tenderness, swelling, or effusion)
Hydrohymenitis	(1) Pleural—chest pain, pleural friction tone, or pleural exudation
Renal lesions	Prominuria > 0.5 g/d or > +++, or cell tube type—it may be of erythrocyte, hemoglobin, granular tube type, or mixed tube type
Nervous system abnormalities	(1) Epilepsy—nondrug or metabolic disorder, such as uremia, ketoacidosis, or electrolyte disorder
Hematological abnormalities	(1) Hemolytic anemia
Immunological abnormalities	(1) Anti-DNA antibody: abnormal titter of anti-double-stranded DNA antibody
Antinuclear antibodies	A positive fluorescent antibody method or equivalent to other tests with abnormal antinuclear antibody titers, ruling out drug-induced “lupus syndrome” (almost all patients with SLE are positive for ANA which is the best indicator for screening for SLE)

**Table 2:** General data of the patients in both groups($\bar{x}\pm s$).

Characteristics	Case group (*n* = 76)	Control group (*n* = 71)
Sex (male/female)	7/69	9/62
Age (age)	37.54 ± 9.68	39.32 ± 5.32
BMI(kg/m^2^)	21.15 ± 3.21	19.71 ± 4.66
Disease course (year)	2.21 ± 4.26	—
SLEDAI (score)	12.60 ± 3.07	—

**Table 3:** The lncRNA expression levels were compared between the different clinical subgroups ($\bar{x}\pm s$).

Groups	lnc0640	lnc3643	lnc5150	lnc7514	lncagf
Arthritis					
+	0.41 ± 0.12	0.92 ± 0.05	0.47 ± 0.20	0.58 ± 0.04	0.37 ± 0.28
-	0.57 ± 0.17	0.83 ± 0.34	0.36 ± 0.21	0.69 ± 0.07	0.28 ± 0.14
Pleuritis					
+	0.58 ± 0.26	0.52 ± 0.43	0.36 ± 0.17	0.34 ± 0.31	0.38 ± 0.10
-	0.57 ± 0.27	0.80 ± 0.31	0.31 ± 0.11	0.63 ± 0.21	0.33 ± 0.15
Erythra					
+	0.56 ± 0.10	0.71 ± 0.52	0.30 ± 0.17	0.53 ± 0.34	0.28 ± 0.19
-	0.53 ± 0.23	0.95 ± 0.76	0.41 ± 0.23	0.60 ± 0.46	0.33 ± 0.14
Myositis					
+	0.42 ± 0.18	0.95 ± 0.45	0.46 ± 0.36	0.54 ± 0.25	0.39 ± 0.17
-	0.54 ± 0.25	0.82 ± 0.46	0.37 ± 0.13	0.74 ± 0.46	0.31 ± 0.11
Fever					
+	0.53 ± 0.18	0.72 ± 0.42	0.39 ± 0.23	0.55 ± 0.32	0.20 ± 0.17
-	0.53 ± 0.25	0.83 ± 0.79	0.48 ± 0.21	0.69 ± 0.32	0.36 ± 0.10

**Table 4:** Analysis of the correlation between the expression level of lncRNAs and laboratory indicators in SLE patients ($\bar{x}\pm s$).

Groups	lnc0640	lnc3643	lnc5150	lnc7514	lncagf
dsDNA					
+	0.41 ± 0.11	0.81 ± 0.04	0.48 ± 0.10	0.48 ± 0.24	0.38 ± 0.18
-	0.48 ± 0.18	0.83 ± 0.34	0.36 ± 0.11	0.68 ± 0.28	0.18 ± 0.14
SM					
+	0.48 ± 0.16	0.41 ± 0.43	0.36 ± 0.18	0.34 ± 0.31	0.38 ± 0.10
-	0.48 ± 0.18	0.80 ± 0.31	0.31 ± 0.11	0.63 ± 0.11	0.33 ± 0.14
SSA					
+	0.46 ± 0.10	0.81 ± 0.41	0.30 ± 0.18	0.43 ± 0.34	0.18 ± 0.18
-	0.43 ± 0.13	0.84 ± 0.86	0.41 ± 0.13	0.60 ± 0.46	0.33 ± 0.14
SSB					
+	0.41 ± 0.18	0.84 ± 0.44	0.46 ± 0.36	0.44 ± 0.14	0.38 ± 0.18
-	0.44 ± 0.14	0.81 ± 0.46	0.38 ± 0.13	0.84 ± 0.46	0.31 ± 0.11
RNP					
+	0.43 ± 0.18	0.81 ± 0.41	0.38 ± 0.13	0.44 ± 0.31	0.10 ± 0.18
-	0.43 ± 0.14	0.83 ± 0.88	0.48 ± 0.11	0.68 ± 0.31	0.36 ± 0.10

**Table 5:** Correlation analysis between lncRNA expression level and SLE disease activity ($\bar{x}\pm s$).

Groups	lnc0640		lnc3643		lnc5150		lnc7514		lncagf	
	rs	*P*	rs	*P*	rs	*P*	rs	*P*	rs	*P*
C4	-0.05	0.32	0.05	0.56	-0.14	0.22	0.05	0.63	-0.07	0.42
ESR	-0.15	0.67	0.46	<0.001	-0.39	0.01	-0.38	<0.001	-0.27	0.02
CRP	-0.12	0.08	0.42	<0.001	-0.15	0.17	-0.25	0.03	-0.02	0.42
DAI score	-0.14	0.54	0.25	0.03	-0.09	0.42	-0.31	0.01	-0.19	0.16
Course of disease	-0.15	0.27	0.19	0.23	0.05	0.60	0.00	0.86	0.09	0.40

## Data Availability

Our data are public and available, and you can query the original data in our database.
